The article "Automated Facial Expression Recognition Framework Using Deep Learning" was published in 2022. Journal: J Healthc Eng.

# Automated Facial Expression Recognition Framework Using Deep Learning

**DOI:** 10.1155/2022/5707930

**Published:** 2022-03-31

**Authors:** Saad Saeed, Asghar Ali Shah, Muhammad Khurram Ehsan, Muhammad Rizwan Amirzada, Asad Mahmood, Teweldebrhan Mezgebo

**Affiliations:** ^1^Faculty of Engineering, Bahria University, Lahore Campus, Lahore, Pakistan; ^2^Faculty of Engineering and Computer Science, National University of Modern Languages, Islamabad, Pakistan; ^3^Department of Electrical and Computer Engineering, Comsats University, Islamabad, Wah Campus, Pakistan; ^4^Ethio Telecom, Addis Ababa, Ethiopia

## Abstract

Facial expression is one of the most significant elements which can tell us about the mental state of any person. A human can convey approximately 55% of information nonverbally and the remaining almost 45% through verbal communication. Automatic facial expression recognition is presently one of the most difficult tasks in the computer science field. Applications of facial expression recognition (FER) are not just limited to understanding human behavior and monitoring person's mood and the mental state of humans. It is also penetrating into other fields such as criminology, holographic, smart healthcare systems, security systems, education, robotics, entertainment, and stress detection. Currently, facial expressions are playing an important role in medical sciences, particularly helping the patients with bipolar disease, whose mood changes very frequently. In this study, an algorithm, automated framework for facial detection using a convolutional neural network (FD-CNN) is proposed with four convolution layers and two hidden layers to improve accuracy. An extended Cohn-Kanade (CK+) dataset is used that includes facial images of different males and females with expressions such as anger, fear, disgust, contempt, neutral, happy, sad, and surprise. In this study, FD-CNN is performed in three major steps that include preprocessing, feature extraction, and classification. By using this proposed method, an accuracy of 94% is obtained in FER. In order to validate the proposed algorithm, K-fold cross-validation is performed. After validation, sensitivity and specificity are calculated which are 94.02% and 99.14%, respectively. Furthermore, the f1 score, recall, and precision are calculated to validate the quality of the model which is 84.07%, 78.22%, and 94.09%, respectively.

## 1. Introduction

A facial expression is to be accounted to know about the emotional state, psychopathology, cognitive activity, and intention of an individual. In interpersonal relations, the facial expressions play an expressive and communicative role. The importance of facial expression recognition (FER) can be gauged from the fact that it can describe any person's mental state or mood. Its applications are not just limited to understand human behaviour, viewing a person's mood, or judging the mental state of humans. It is also penetrating into other fields such as criminology, holographic, smart healthcare systems, security systems, education, robotics, entertainment, multimedia communication, and stress detection [1–7]. The integration of facial expressions in these fields shows that facial expressions have an essential part in human life. Automatic FER is presently one of the most challenging tasks in the field of computer sciences. Expressions can be conveyed through gestures and communications. It does not just depend on the human face. Mehrabian et al. [8] say that a person can transfer only 7% of the information context orally, while 38% can be transferred through voice tone, rhythm, and how speedily or slowly a person speaks. On the other hand, the information which is transferred through facial expressions is 55%. Through facial expression, one can understand the mental state of the other person. Ekman et al. [9, 10] introduced the facial emotions into seven basic categories which include happy, fear, sad, surprise, anger, contempt, and disgust.

The article "Automated Facial Expression Recognition Framework Using Deep Learning" was published in 2022. Journal: J Healthc Eng.

Applications of facial expressions cover a huge area of our society and are not just limited to some specific fields. In medical sciences, FER is beneficial for bipolar patients. As described in [11], doctors are trying to detect and monitor patients' behavior, such as how a bipolar patient feels and how they behave during their disease. In [12], an intelligent FER system is devised such that facial images are given as input and the system can detect the expressions of a human face. There are in total 8 expressions [13, 14] that a human can express which include fear, happy, surprise, neutral, angry, contempt, sad, and disgust state.

In this study, the eight expressions are used, and an algorithm named FD-CNN is proposed to improve the accuracy of FER. Three major building blocks: preprocessing, feature extraction, and classification are further categorized to obtain the underlying objective. In this process of FER, the extended Cohn-Kanade (CK+) dataset is chosen. It has images extracted from 123 different people, including males and females. All images are captured from the front angle and divided into eight different categories. In the first phase of preprocessing, all the images are reshaped to 150 × 150 pixels so that all images have an equal size. Further, in preprocessing, images are randomly rotated between 0 and 180 degrees and zoomed. Images are also flipped horizontally and vertically. In the next phase, images are further processed to extract features. In feature extraction, a filter or kernel is applied to the image, and this kernel can be of different sizes according to the required features. In this study, 3 × 3 kernel is used to address the tradeoff between the feature extraction requirements and computation cost. After applying the said sized kernel, the output comes out in the form of face curves and edges. Once the features are extracted, then there is a need to keep only useful features, and max pooling helps out in this regard. Classification is the third phase of the proposed methodology, and it is responsible for detecting the correct labels. In classification, fully connected layers are used, and these fully connected layers use two hidden layers further. Each hidden layer has multiple nodes that have some weights. There is a process called forward propagation in which the weight to these nodes are multiplied with bias values and then summed up all. In backpropagation, the weight of the hidden layer's nodes is adjusted, and the model can find the true label of an input image.

The article "Automated Facial Expression Recognition Framework Using Deep Learning" was published in 2022. Journal: J Healthc Eng.

The remaining part of this paper is organized as follows: in Section 2, the state-of-the-art-work of FER is described.  Section 3 discusses the methodology of the proposed algorithm in detail. Simulations and results are described in Section 4. In the end, the presented work is concluded in Section 5.

## 2. Literature Review

Facial expressions play a crucial role in our everyday life while communicating with others. In 1978, the first ever automatic FER system was introduced by Suwa [15], in which he explained how he identified 20 spots in an image sequence to find facial expressions.

Pantic and Rothkrantz [16] proposed a system for automatic recognition of facial gestures from a static coloured face image. They employed the multidetector technique for facial feature localization to combine facial regions' contours and profile contours like eyes and mouth. Using rule-based reasoning, the author extracted 10 fiducial points of the profile contour and 19 fiducial points of the facial component contours, while 32 facial muscle action units [17] were recognized with 86% accuracy.

Chen et al. [18] proposed a system for facial expression using a hybrid method based on geometric and appearance features that found the difference of points from a neutral facial image and an emotional facial image. This hybrid feature contains the local texture difference and the facial feature point displacement. The accuracy of the proposed method is 95% on the CK + database by using the support vector machine (SVM) classifier.

Uçar et al. [19] proposed a methodology for FER by using the curvelet transform (CT) and the online sequential extreme learning machine (OSELM) with a radial basis function. In the first step, the face is divided into some small regions which are called local regions, and then the CT is smeared to that local region of the face. The main purpose of doing this is to reduce the curvelet coefficients so that they can be easily classified within a minimum time. Furthermore, they calculated the standard deviation, entropy, and mean of curvelet coefficient to generate the set of features for each region. To increase the classification and reduce the time required in choosing the hidden node number, they used the spherical clustering method on the feature set. The learning is then called OSELM-SC and it consists of two parts. The first part checks the performance of OSELM-SC on different datasets, and the second part tests the accuracy of the FER algorithm on the Japanese Female Facial Expressions (JAFFE) and Cohn Kanade (CK) database.

The article "Automated Facial Expression Recognition Framework Using Deep Learning" was published in 2022. Journal: J Healthc Eng.

One of the challenging tasks for accurate FER is the extraction of emotional features correctly from the input images. In [20], salient distance features are used to solve the problem of extracting facial features accurately, while these salient features are obtained by extracting patch-based 3D Gabor features. The results show that the good CRR, i.e., the correct recognition rate and the system performance, is improved by considering the facial and muscle movements. They get a good accuracy rate by using the JAFFE and CK databases.

In [21], a kernel-based manifold learning method is proposed, which is called KDIsomap, i.e., kernel discriminant isometric mapping. KDIsomap extracts the discriminant information nonlinearly. It is also used as a dimensionality reduction on extracted facial features. They use the closest neighbor classifier to the Euclidean metric to recognize facial expressions. This classifier is applied to two publicly available databases, which are JAFFE and CK. Using KDIsomap, the obtained accuracy is 94.88% on the CK database and 81.59% accuracy is obtained on the JAFFE database.

In human-computer interaction, FER plays a crucial role. Jabid et al. [22] presented the appearance-based feature descriptor, which is, i.e., local directional pattern (LDP). This LDP represents the facial geometry and evaluates FER performance. In each pixel, by computing the edge response values, LDP features are obtained. These features are then encoded into an 8-bit binary number. Principal component analysis (PCA) and AdaBoost are then used for dimensionality reduction, which in turn benefits us with less computation and better classification accuracy. Template matching and SVM are two machine learning methods that are applied to CK and JAFFE databases to recognize facial expressions.

The article "Automated Facial Expression Recognition Framework Using Deep Learning" was published in 2022. Journal: J Healthc Eng.

Negative emotional states can cause a mental health problem. So, to improve people's health, especially for the elderly, Uddin et al. [23] proposed an efficient method for the FER which is helpful in emotional healthcare systems. In the proposed FER, a video data is used to detect the facial states of human, also the feature extraction is employed to extract the predominant features from the given dataset. For robust feature extraction, the local directional position pattern (LDPP) method is used. Furthermore, they used PCA and generalized discriminant analysis (GDA), respectively, to reduce the selected features, and these features were then used in the deep belief network (DBN) for the FER.

In [24], they used an extensive range of head postures for FER. Their methodology, mapped the nonfrontal view features with the corresponding features of the frontal view within the same facial expression. For FER, they first estimated the posture of the head in the given input image and then applied mapping. The extracted features after mapping were very trustworthy for recognition purposes. The authors evaluated their results by applying the methods on multi-PIE and BU3DFE datasets, and good results were achieved.

In [25], the authors tried to do local learning for FER in which they used a convolutional neural network (CNN) for automatic feature learning and a bag of visual words (BOVW) model is used for handcrafted feature learning. These two types of features are combined to find out the best result of FER. There are three steps for the local learning framework which are used in the paper. First, K nearest neighbour (KNN) is used to select only those images from the training data that are closest to the input test image. Secondly, SVM is trained using selected images and then, based on that training, SVM classifies the input test images efficiently. In this research, the authors used 4 different datasets which are FER 2013, FER+, AffectNet with eight expressions, and AffectNet with seven expressions. The accuracies of the proposed method with said datasets are 75.42%, 87.76%, 59.58%, and 63.31%, respectively.

In [26], automatic FER is performed by using occlusion and pose variation. The authors used the real-world FER dataset with different poses and occlusion attributes, and the method that was used is region attention network (RAN). They validated RAN using four different datasets named as SFEW, RAF-DB, AffectNet, and FER Plus. The obtained accuracies are 56.4%, 86.9%, 59.5%, and 89.16%, respectively.

The article "Automated Facial Expression Recognition Framework Using Deep Learning" was published in 2022. Journal: J Healthc Eng.

## 3. Dataset

In this study, the dataset used is CK + as detailed in Table 1. This dataset is obtained from the Kaggle dataset website. The images consist of 640 × 490 pixels from 123 different human faces including males and females.

There are 920 images in total which are used in this research for training and testing of the proposed FD-CNN. These images are labeled with eight emotions including fear, happy, sad, contempt, disgust, neutral, surprise, and anger, as shown in Figure 1. All these images are captured from the front angle.

## 4. Methodology

The methodological framework is pictorially presented in Figure 2. The methodology consists of preprocessing, feature extraction, and classification that are discussed as following.

Figure 2 shows that the acquired dataset is preprocessed at the first phase of the proposed framework FD-CNN. This FD-CNN uses CNN with four convolutional layers and two hidden layers. Once preprocessing is completed, information is passed to the next phase called feature extraction. In the feature extraction phases, many substages help to extract features, and only valuable features are kept for further processing. In the end, classification is performed to recognize label of the input image correctly. To find the correct label of the input image, forward and backward propagation are exploited for error estimation and minimization.

### 4.1. Preprocessing

Preprocessing is used to improve the system performance by transforming the inconsistent dataset into a consistent dataset. Consistency is obtained by reshaping all the images into 150 × 150 pixels. Further, in this step, all images are randomly rotated between 0 and 180 degrees, and they are also zoomed randomly. Images are also flipped horizontally and vertically too.

### 4.2. Architecture of CNN

CNN is one of the conventional forms of deep neural networks. It takes images as input, and with the help of learnable weights and biases, it can differentiate in different images. These weights and biases are used in hidden layers. CNN is mostly used for analyzing visual imagery [27, 28].

Main building blocks of CNN include feature extraction and other one is classification. Feature extraction is further subdivided into convolution, padding, nonlinearity, and pooling. In CNN, classification contains a fully connected layer [29], as shown in Figure 3. This fully connected layer is made up of hidden layers, and one hidden layer contains many neurons. Each neuron in a layer is linked to all the neurons in the next hidden layer [30].

### 4.3. Feature Extraction

Feature extraction is performed to find out the useful information which is exploited for the classification of images. For example, if we have an image of a human face, then through feature extraction, we can find out the eyes, nose, and lips of the input human face [31]. Feature extraction has further substages which are explained as following.

The article "Automated Facial Expression Recognition Framework Using Deep Learning" was published in 2022. Journal: J Healthc Eng.

#### 4.3.1. Convolution

Convolution is performed on an input image by using a filter or a kernel in CNN. The kernel used in this paper is 5 × 5 in size. In order to perform this filtering and convolution, we do a scan of the whole image [32]. We start scanning from the top left side of the image and go to the right side and then move one bit down and repeat the same procedure from left to right until the whole image is scanned.

#### 4.3.2. Padding

Padding can be categorized as valid padding or same padding [33]. In valid padding, the dimensionality is to be reduced from the original one, while in same padding, the dimensionality is either to be increased or remain the same as compared to the original one, depending on the case or situation [34]. In the proposed FD-CNN, the same padding is used, in which the dimensionality is to remain same.

#### 4.3.3. Nonlinearity

After moving our filter from top left to right on our original input image, the resultant output will pass through one more step called a nonlinearity function or activation function. This activation function is called ReLu the Rectified Linear Unit and it is mainly used in CNN for feature extraction [35]. The working of this ReLu function is so simple. It just converts all the negative values of the matrix into 0 and does not change the positive values.

#### 4.3.4. Pooling

Once you get the feature map from the convolutional layer, it is time to add a subsampling layer or pooling in CNN layers. Just like the convolutional layer, the pooling layer also reduces the size of the convolved features [36]. After the dimensionality reduction, there is less computational power required to process the data. Pooling is very helpful for extracting features from those images which are rotational and positional invariant. Pooling is also helpful in shortening the training time and controlling overfitting.

There are two types of pooling which can be applied [37]. The first one is max pooling, and the other one is average pooling. In max pooling, it returns the maximum value from a region where the kernel or filter overlaps with the input image. In average pooling, the average of the values from the region where kernel overlaps with the input image is returned. In this FD-CNN, we used max pooling. The reason behind choosing it is that max pooling avoids noise from the image in the calculation because it takes the maximum value from the selected region, while in average pooling noise can be added because it takes the average of the whole region.

The article "Automated Facial Expression Recognition Framework Using Deep Learning" was published in 2022. Journal: J Healthc Eng.

#### 4.3.5. Fully Connected Layer

In the CNN, there are two hidden layers, and each hidden layer contains different sets of neurons. Each neuron is fully connected with the neurons of the next layer [38]. In this network, the information comes from the feature extraction and is used in the hidden layer where the output values come from the multiplication of each neuron weight with bias value [39], then the summation of these obtained values is compared with the actual output value, and this process is called forward propagation [40]. If our calculated value is not nearest to the actual value, then the weights of neurons are adjusted, and this process is called backpropagation [41]. In the end, when the required output value is gained by using backpropagation, the model then classifies the input images and labels them according to the obtained values.

## 5. Simulation and Results

The proposed model implementation is also validated by using different tests. These tests include independent tests, K-fold cross-validation, the confusion matrix, recall, precision, F1 measure, and the ROC curve. This study calculates the system's sensitivity and specificity, and the results are to be discussed.

### 5.1. Evaluation

In order to validate the performance of FD-CNN, 10-fold cross validation test is performed. The confusion matrix, sensitivity, and specificity of the FD-CNN are then evaluated.

### 5.2. Independent Test Set

In the independent test, the dataset is segregated into training and testing by an 8 : 2 split ratio, but this split ratio can be changed according to the needs. After that, the proposed model is trained using a training dataset and the model is validated using a test dataset. The CNN classifier is used for the classification of images into eight categories, and the accuracy of FD-CCN is evaluated. Besides the precision, the recall f1 score, sensitivity, and specificity are calculated.

#### 5.2.1. Confusion Matrix

The CK + dataset is used to train and validate the FD-CNN. A confusion matrix of the FD-CNN is obtained, as shown in Table 2. It contains the eight classes of facial emotions that include surprise, sad, neutral, happy, fear, disgust, contempt, and anger.

In Table 2, the rows show the actual classes, and the columns show the predicted classes. According to the confusion matrix, the results describe that the model efficiently predicts the classes of disgust, happy, neutral, and surprise with high accuracy of 82%, 100%, 100%, and 89%, respectively. Anger, contempt, and fear classes are predicted with 29%, 33%, and 25% accuracy, respectively. In contrast, a sad class is predicted with satisfactory results. The confusion matrix also shows that the anger class is misclassified as 43% disgust and 29% neutral. The contempt class is 67% misclassified as neutral. Disgust and fear are also misclassified. In the case of disgust, it is misclassified as 12% anger and 6% neutral, whereas fear is misclassified as 25% disgust and 50% neutral. Similarly, sad and surprise are misclassified. In the case of sad it is misclassified as 17% anger, 17% contempt, 33% neutral, and 17% surprise whereas surprise is misclassified as 11% neutral only.

The article "Automated Facial Expression Recognition Framework Using Deep Learning" was published in 2022. Journal: J Healthc Eng.

In Table 3, all the true and predicted values of confusion matrix for 100 epochs with data duplication are shown.

Data duplication increases the size of the dataset, and with the increase of the dataset, the model can train itself better. Table 3 shows eight rows and eight columns of emotion, while the rows show the actual classes and the columns show the predicted classes. According to the confusion matrix, the results validate that the model efficiently predicts the classes of anger, contempt, disgust, fear, happiness, neutral, and surprise with high accuracy of 94%, 94%, 100%, 90%, 100%, 100%, and 100%, respectively. Anger and contempt classes are predicted with 94% and 94% accuracy, but misclassified with 6% disgust in the case of anger and 6% neutral in the case of contempt. In comparison, fear classes are predicted at 90% but misclassified with 10% neutral class. The sad class is only predicted 86% correct and easily misclassified with 14% neutral class.

Table 4 shows all the true and predicted values of confusion matrix for 1000 epochs.

According to the confusion matrix in Table 4, the results describe that the model efficiently predicts the classes of disgust, happiness, neutral, and surprise with high accuracy of 94%, 100%, 99%, and 94%, respectively. Anger and contempt classes are predicted with an accuracy of 71% and 67%, respectively. At the same time, fear and sad classes are predicted with satisfactory results. The confusion matrix also shows that the anger class is misclassified as 14% disgust and 14% neutral. Contempt is misclassified as 33% neutral. Disgust and fear are also misclassified; in the case of disgust, it is misclassified as 6% neutral, whereas fear is misclassified as 25% disgust and 25% neutral. Similarly, sad and surprise are misclassified; in the case of sad, it is misclassified as 33% neutral and 17% surprise, whereas it is misclassified as 6% neutral only in the case of a surprise. The neutral class is just 1% misclassified as sad. The low accuracy of fear and sadness compared to others is due to the smaller number of images of these classes. As the information is not well sufficient to train the model, accuracy will also be compromised.

The article "Automated Facial Expression Recognition Framework Using Deep Learning" was published in 2022. Journal: J Healthc Eng.

#### 5.2.2. Model Loss

A model loss is a metric to penalize the model if it does not correctly predict the input data. The loss of the proposed FD-CNN is shown for 100 epochs without data duplication in Figure 4. While in Figure 5, loss of the FD-CNN is shown for 100 epochs with data duplication.

Figure 6 shows the FD-CNN loss for 1000 epochs without data duplication.

#### 5.2.3. Model Accuracy

The training and testing accuracy of FD-CNN for 100 epochs is shown in Figure 7 without data duplication. While the accuracy of FD-CNN for 100 epochs with data duplication is shown in Figure 8.

Figure 9 shows the FD-CNN accuracy for 1000 epochs without data duplication.

In order to validate the performance of the proposed methodology, a 10-fold cross validation is also performed. In 10-fold cross validation, the dataset is shuffled randomly and then divided into ten equal folds. In every iteration, a unique fold is taken as test data and the remaining folds as training data. After training, FD-CNN is validated using a test fold with a certain accuracy. When all 10 folds are performed, the obtained accuracies are summed up and their average is taken to calculate the final score of the accuracy, as shown in Table 5.

#### 5.2.4. Evaluation through Precision, Recall, and F1 Score

The quality of a proposed model FD-CNN is to be evaluated with measured recall, precision, and f1 score. These metrics help in better classification of multiclassification problems, as shown in Table 6.

#### 5.2.5. Sensitivity and Specificity

The sensitivity and specificity of FDD-CNN are estimated with and without data duplication. The estimated metrics are presented in Table 7. The sensitivity evaluates the model's capability to predict true positives while specificity evaluates the model's capability to predict true negatives of every available category in the dataset, respectively.

#### 5.2.6. Receiver Operating Characteristic (ROC) Curve

The ROC curve is used to evaluate the performance of multiclassification problems at different thresholds and, with ROC, the term area under the curve (AUC) is also frequently used. The ROC curve shows how well the given model is performing at each point. If AUC is higher, it shows that the given model is correctly predicting the available classes in the dataset under test; otherwise, it represents the inefficiency of the given model under the given scenario. The ROC curves of the proposed FD-CNN for 100 epochs without data duplication and with data duplication are shown in Figures 10 and 11, respectively. While in Figure 12, the ROC of the FD-CNN is shown for 1000 epochs without data duplication. The higher AUC shows the comparatively good performance of the proposed FD-CNN.

The article "Automated Facial Expression Recognition Framework Using Deep Learning" was published in 2022. Journal: J Healthc Eng.

### 5.3. Comparison of Results

The comparison of the proposed FD-CNN with the state-of-the-art work intelligent FER frameworks using deep learning techniques is described in Table 8.

In Table 8, it is shown that the framework proposed by Georgescu et al. [25] achieved 87.76% and the learning model proposed by Nianyin et al. [42] achieved 89% accuracy by considering the dataset CK+ with duplication of data for 100 epochs. The proposed model FD-CNN with the same CK + dataset obtained an accuracy of 89.13% without duplication of data while 97% with duplication of data for 100 epochs, as did in [25, 42].

There are two major reasons for selecting [25, 42] to have a comparison. First one, the authors used the CK + dataset, and the other one is that deep neural network is used in both proposed frameworks. Specifically, in [42], the author used the DSAE model to train its dataset. DSAE is from a family of deep neural networks. In this research work, CNN is used, which belongs to the deep neural network family and trains the model on the training dataset. To classify the images of the input dataset, [42] used the softmax classifier while in our proposed work, the softmax classifier is used to predict the true labels of images based on training. DSAE extracted the useful information from the input images, and the softmax classifier used this information for classifying the images among different categories. In the DSAE architecture, four layers are used in total. The first one is the input layer, the second and third are the hidden layers, and the fourth is the output layer. While in our proposed study, four convolutional layers, two hidden layers and one output layer are used. In [42], the features are extracted by using the histogram of oriented gradients (HOG) and these features are reduced with PCA. The model is then trained based on these features. While in our proposed FD-CNN, ReLu is used for the features that are to be extracted. Both studies are using backpropagation to fine-tune the model by minimizing the error rate. The total number of images of the CK + dataset with duplication used in [42] is 1635, while a total of 920 images of CK + without duplication and 1635 images with duplication are used in our proposed framework. For validation purposes, 10-fold cross-validation is used to evaluate the performance of the proposed model by measuring the parameters like sensitivity, specificity, precision, recall, and f1 measure.

## 6. Conclusions

In this study, an algorithm FD-CNN with four convolutional layers and two hidden layers is proposed for automatic FER to improve accuracy. Facial expression detection through facial images is used in many applications, including smart healthcare systems, criminology, holographic, security systems, education, robotics, entertainment, and stress detection. Compared to the previous work, where mostly six or seven expressions are used with different types of neural network. This research work used eight expressions for facial expression recognition. In this proposed method, the CK + dataset is used, with 123 different people, including males and females, with expressions such as anger, fear, happiness, sadness, disgust, contempt, neutral, and surprise. The proposed FD-CNN consists of preprocessing, feature extraction, and finally classification. In preprocessing, images are reshaped to 150 × 150 so that all images have an equal size. Furthermore, images are rotated randomly between 0 and 180 degrees, zoomed horizontally, and flipped vertically. After preprocessing, FD-CNN is used to extract the essential features. These extracted features are then used to classify facial expressions and send to the fully connected layer. Where through forward propagation, the error rate is estimated, and this error is then minimized by using backpropagation. In the end, the CNN classifier gives the label to these images based on the weighted score. The obtained accuracy of FDD-CNN for 100 epochs with data duplication is better than the state of the artwork as mentioned in the previous section.

The article "Automated Facial Expression Recognition Framework Using Deep Learning" was published in 2022. Journal: J Healthc Eng.

The FD-CNN algorithm is also validated by using 10-fold cross-validation to validate its performance. This validation test includes precision, recall, and the f1 measure which is 94.09%, 78.22%, and 84.07%, respectively. Furthermore, the calculated sensitivity and specificity are 94.02% and 99.14%, respectively.

## Figures and Tables

**Figure 1:** Eight emotions of CK + dataset.

**Figure 2:** Methodology.

**Figure 3:** Architecture of the convolutional neural network.

**Figure 4:** Model loss for 100 epochs.

**Figure 5:** Model loss for 100 epochs with data duplication.

**Figure 6:** Model loss for 1000 epochs.

**Figure 7:** Model accuracy for 100 epochs.

**Figure 8:** Model accuracy for 100 epochs with data duplication.

**Figure 9:** Model accuracy for 1000 epochs.

**Figure 10:** ROC curve for 100 epochs.

**Figure 11:** ROC curve for 100 epochs with data duplication.

**Figure 12:** ROC curve for 1000 epochs.

**Table 1:** Metadata for dataset.

Sr. No	Emotions	Number of emotions
1	Anger (An)	45
2	Contempt (Co)	18
3	Disgust (Di)	59
4	Fear (Fe)	25
5	Happy (Ha)	69
6	Neutral (Nu)	593
7	Sad (Sa)	28
8	Surprise (Su)	83

**Table 2:** Confusion matrix for 100 epochs.

	An	Co	Di	Fe	Ha	Ne	Sa	Su
An	29%	0	43%	0	0	29%	0	0
Co	0	33%	0	0	0	67%	0	0
Di	12%	0	82%	0	0	6%	0	0
Fe	0	0	25%	25%	0	50%	0	0
Ha	0	0	0	0	100%	0	0	0
Ne	0	0	0	0	0	100%	0	0
Sa	17%	17%	0	0	0	33%	17%	17%
Su	0	0	0	0	0	11%	0	89%

The article "Automated Facial Expression Recognition Framework Using Deep Learning" was published in 2022. Journal: J Healthc Eng.

**Table 3:** Confusion matrix for 100 epochs with data duplication.

	An	Co	Di	Fe	Ha	Ne	Sa	Su
An	94%	0	6%	0	0	0	0	0
Co	0	94%	0	0	0	6%	0	0
Di	0	0	100%	0	0	0	0	0
Fe	0	0	0	90%	0	10%	0	0
Ha	0	0	0	0	100%	0	0	0
Ne	0	0	0	0	0	100%	0	0
Sa	0	0	0	0	0	14%	86%	0
Su	0	0	0	0	0	0	0	100%

**Table 4:** Confusion matrix for 1000 epochs.

	An	Co	Di	Fe	Ha	Ne	Sa	Su
An	71%	0	14%	0	0	14%	0	0
Co	0	67%	0	0	0	33%	0	0
Di	0	0	94%	0	0	6%	0	0
Fe	0	0	25%	50%	0	25%	0	0
Ha	0	0	0	0	100%	0	0	0
Ne	0	0	0	0	0	99%	1%	0
Sa	0	0	0	0	0	33%	50%	17%
Su	0	0	0	0	0	6%	0	94%

**Table 5:** Model accuracy.

Tests	Dataset	Accuracy (%)
Independent test set for 100 epochs	CK+	89.13
Independent test set for 100 epochs with data duplication	CK+	97
Independent test set for 1000 epochs	CK+	94
10 fold cross validation for 100 epochs	CK+	95.85
10 fold cross validation for 100 epochs with data duplication	CK+	99.79
10 fold cross validation for 1000 epochs	CK+	98.64

**Table 6:** Classification report.

Tests	Precision (%)	Recall (%)	F1 score (%)
Independent test set for 100 epochs	81.67	59.35	63.61
Independent test set for 100 epochs with data duplication	98.40	95.54	96.82
Independent test set for 1000 epochs	94.09	78.22	84.07
10 fold cross validation for 100 epochs	78.1	81	78.8
10 fold cross validation for 100 epochs with data duplication	99.10	98.40	98.40
10 fold cross validation for 1000 epochs	85.5	86.9	85.9

**Table 7:** Sensitivity and specificity.

Tests	Parameters	Results (%)
Independent test set for 100 epochs	Sensitivity	86.95
	Specifity	98.68
Independent test set for 100 epochs with data duplication	Sensitivity	97.55
	Specifity	99.69
Independent test set for 1000 epochs	Sensitivity	94.02
	Specifity	99.14
10 fold cross validation for 100 epochs	Sensitivity	83.28
	Specifity	97.63
10 fold cross validation for 100 epochs with data duplication	Sensitivity	99.17
	Specifity	99.88
10 fold cross validation for 1000 epochs	Sensitivity	94.53
	Specifity	99.22

**Table 8:** Comparison of Results

Dataset	Georgescu et al.	Nianyin et al.	FD-CNN
CK+	87.76%	89%	94%

## Data Availability

The data are available from the following link: https://paperswithcode.com/dataset/ck.
